The article "Non-human Primate Regulatory T Cells and Their Assessment as Cellular Therapeutics in Preclinical Transplantation Models" was published in 2021. Journal: Front Cell Dev Biol.

# Non-human Primate Regulatory T Cells and Their Assessment as Cellular Therapeutics in Preclinical Transplantation Models

**DOI:** 10.3389/fcell.2021.666959

**Published:** 2021-06-15

**Authors:** Angus W. Thomson, Kazuki Sasaki, Mohamed B. Ezzelarab

**Affiliations:** ^1^Department of Surgery, Thomas E. Starzl Transplantation Institute, University of Pittsburgh School of Medicine, Pittsburgh, PA, United States; ^2^Department of Immunology, University of Pittsburgh School of Medicine, Pittsburgh, PA, United States

**Keywords:** regulatory T cells, non-human primates, transplantation, cell therapy, immunobiology

## Abstract

Non-human primates (NHP) are an important resource for addressing key issues regarding the immunobiology of regulatory T cells (Treg), their *in vivo* manipulation and the translation of adoptive Treg therapy to clinical application. In addition to their phenotypic and functional characterization, particularly in cynomolgus and rhesus macaques, NHP Treg have been isolated and expanded successfully *ex vivo*. Their numbers can be enhanced *in vivo* by administration of IL-2 and other cytokines. Both polyclonal and donor antigen (Ag) alloreactive NHP Treg have been expanded *ex vivo* and their potential to improve long-term outcomes in organ transplantation assessed following their adoptive transfer in combination with various cytoreductive, immunosuppressive and “Treg permissive” agents. In addition, important insights have been gained into the *in vivo* fate/biodistribution, functional stability, replicative capacity and longevity of adoptively-transferred Treg in monkeys. We discuss current knowledge of NHP Treg immunobiology, methods for their *in vivo* expansion and functional validation, and results obtained testing their safety and efficacy in organ and pancreatic islet transplantation models. We compare and contrast results obtained in NHP and mice and also consider prospects for future, clinically relevant studies in NHP aimed at improved understanding of Treg biology, and innovative approaches to promote and evaluate their therapeutic potential.

## Introduction

NHP are a valuable resource for translational research on innovative therapies with potential for clinical application. These include strategies to promote transplant tolerance without the toxicities and morbidities associated with immunosuppressive (IS) drugs that fail to induce clinical tolerance (Knechtle et al., 2019). Mouse models of tolerance induction are inadequate predictors of tolerance in both NHP and humans (Sachs, 2003). This reflects the fact that unlike the latter species, specific pathogen-free (spf) laboratory mice do not acquire heterologous immunity, i.e., virus-induced T cell memory that constitutes a powerful barrier to tolerance induction (Adams et al., 2003). In addition, whereas MHC class II Ags that are key to induction of alloimmunity are absent from rodent vascular endothelium, they are expressed constitutively by these cells in large animals (Choo et al., 1997; Houser et al., 2004). Due to (i) similarities between NHP and human immune systems, (ii) cross-reactivity between drug targets in these species, (iii) the outbred nature of NHP, (iv) their natural exposure to environmental pathogens, and (v) their longevity compared with mice, NHP are important models for studying mechanisms underlying immune regulation and tolerance (Fitch et al., 2019). NHP also allow evaluation of the scalability and safety of innovative therapeutic strategies (e.g., monitoring and management of adverse events, such as potential infusion reactions and infectious complications) and associated techniques, e.g., leukapheresis in conjunction with cell therapy, that are not practiced in rodents.

NHP Treg phenotype and function resemble those of human Treg (Anderson et al., 2008; Haanstra et al., 2008). As in humans, testing of their efficacy is dependent on their isolation, massive expansion and product validation. The ability to assess the *in vivo* stability and migration of adoptively-transferred Treg is also an important translational aspect of studies of these cells in NHP and crucial for their assessment as cellular therapeutics.

## Isolation, Purification, *ex vivo* Expansion and Validation of NHP Treg

Details of methods developed for isolation and purification of NHP Tregs from blood or tissues, and for expansion and testing of polyclonal, polyspecific or donor Ag-alloreactive (dar) NHP Treg are summarized in Table 1. Thus, *ex vivo* expansion of cynomolgus or rhesus Treg after immunomagnetic bead or/and flow sorting has been well-described in response to either polyclonal stimuli (Gansuvd et al., 2007; Anderson et al., 2008), allogeneic PBMC (Porter et al., 2007) or dendritic cells (DCs) (Moreau et al., 2008), artificial (a)APCs (Weiner et al., 2015; Zhang et al., 2015) or CD40L-stimulated allogeneic B cells (sBc) (Ezzelarab et al., 2020; Alonso-Guallart et al., 2021). Most recent attention has focused on expansion of alloreactive Tregs using various protocols. Thus, Alonso-Guallart et al. (2021) expanded highly suppressive cynomolgus polyspecific Tregs using a combination of CD40L−engineered B cells from 3 to 4 animals representative of diverse MHCs. The expanded Tregs expressed high levels of Foxp3 and Helios, a high incidence of Treg-specific demethylated region demethylation, and markedly suppressed naïve T cell responses *in vitro*. Importantly, these Tregs also expanded after cryopreservation, an important benefit allowing protocol flexibility. Specificity assays confirmed they were suppressive following activation by any APCs whose MHC expression was shared by the CD40L−sBc used during their expansion, proving that they were polyspecific (Alonso-Guallart et al., 2021). Recently, Ezzelarab et al. (2020) also used CD40L−sBc of donor origin to expand cynomolgus darTregs that were adoptively-transferred to transplant recipients.

**TABLE 1:** Timeline of reports of Treg isolation, expansion and suppressive activity in NHP species.

Species	Treg selection (purity)	Cell yield	Expansion method	Expansion rate	Suppressive activity	Reference(s)
Rhesus macaque	T cells from spleen	200 × 10^6^ cells per recipient (splenectomized)	Donor splenocytes + anti-CD80/CD86; 13 days	2–4-fold	*In vivo* infusion 13 days post allogeneic kidney transplant; donor-specific inhibition of rejection	Bashuda et al., 2005
Rhesus	MACS (90%) or FACS (98%) CD4^+^ CD25^+^	Not indicated	Anti-CD3/CD28 beads + IL-2; 4 weeks	300–2,000-fold	Up to 1:8^*a*^ ratio, suppression of autologous PBMC proliferation	Gansuvd et al., 2007
Rhesus	Anti-CD8 and anti-CD20 Dynabeads, or CD4^+^ MACS, followed by anti-CD25 MACS (82%)	10% of CD3^+^CD4^+^ T cells	Fresh cells used; no expansion	n/a	Proliferation of Teff in response anti-CD3 or irradiated PBMC decreased at 1:1^*a*^ ratio, however variation between animals	Haanstra et al., 2008
Rhesus	FACS CD4^+^CD25^*hi*^ or CD4^+^CD25^+^CD127^–^	10^5^ cells/mL blood	Anti-CD3/CD28 beads + IL-2; 4 weeks	Up to 450-fold	CFSE-MLR, up to 1:100^*a*^ ratio; suppression of alloreactive response by responder-specific or third-party Treg	Anderson et al., 2008
Rhesus	MACS CD4^+^CD127^–/lo^	7% of CD4^+^/1.3% of total PBMC; 3.7 × 10^4^ cells/ml blood	Immature Mo-DC^+^ IL-2^+^ IL-15; 14 days, or 10 days followed by 2 days without DC	No expansion	Suppression up to 1:40^*a*^ ratio; donor-specific	Zahorchak et al., 2009
Rhesus	FACS CD4^+^ CD25- CD127^–^/lo cells (> 80%)	>or = 10^6^	Stimulation with anti-CD3 and anti-CD28 microbeads (1 cell: 2 beads) + IL-2 (2,000 U/ml) ± rapamycin (1,000 nM); re-stimulation at 7 and 14 days; harvested on day 21	210–760-fold	Strong suppression of CD4^+^ and CD8^+^ T cell proliferation in CFSE-MLR	Singh K. et al., 2012
Cynomolgus macaque	FACS CD4^+^ CD25^+^CD127^–^ (> 98%)	0.4% of PBMC	Allo DC (BM-DC/Mo-DC) + IL-2; 7 days	12–25-fold	CFSE-MLR, PBMC^+^ anti-CD3/CD28^+^ Treg: 30% inhibition at 1:3^*a*^ ratio. Treg suppressive function stimulated by BM-DC > Mo-DC	Moreau et al., 2008
Cynomolgus (MS model)	MACS CD4^+^ CD25^+^ (>90%)	6.4% of T cells	Fresh cells used; no expansion	n/a	Proliferation to anti-CD3/CD28 or CD3/CD46 stimulation impaired during active MS	Ma et al., 2009
Cynomolgus	FACS CD4^+^CD25^*hi*^CD127^–^ from PBMC	5% total CD4^+^ cells	NHP-specific anti-CD2/3/28 microbeads (cell: bead ratio 1:2), rhu IL-2 (1,000 U/ml) and rhu TGF-b; 5 ng/mL); 20 day culture	>80-fold	Strong suppressive effect at ratios up to 1:4 (Treg:Teff) on CD4^+^ and CD8^+^ T cell proliferation	Dons et al., 2013
Cynomolgus	FACS CD4^+^CD25^+^CD127^–^ (>95%)	4.7 (2–6.9)% of blood CD4^+^ cells	Artificial (a)APCs (L32) loaded with anti-CD3 (1:1 ratio) for 7–8 days with IL-2 + rapamycin; restimulation with aAPCs on days 7 and 14 without rapamycin; harvested on day 21	1,000-fold	Potent suppression of anti-CD3/CD28-indiced CD4 and CD8 T cell proliferation	Guo et al., 2015; Zhang et al., 2015
Cynomolgus	FACS CD4^+^CD25^*hi*^CD127^*lo*^	0.5–1% of total PBMC	Donor Ag alloreactive Tregs stimulated with donor CD40L-activated B cells + IL-2; harvest on day 9 and co-culture with aAPCs (L32 cells) + IL-2 for 2 subsequent rounds of 7 days	10,000-fold	Strong suppression (>polyclonal Tregs) of autologous T cell proliferation in MLR in response to donor APCs.	Ezzelarab et al., 2020
Cynomolgus	FACS CD4 + CD8^–^CD25^*hi*^CD127^–^	Top 1% CD25^+^ cells in the CD4^+^ CD8^–^CD127^–^ gate	Polyspecific Tregs expanded with a panel of CD40L-stimulated B cells (CD40L−sBc)	10,000-fold after 28 days (4 rounds)	Expanded Tregs suppressive after activation by any APCs whose MHC was shared by CD40L−sBc used during expansion	Alonso-Guallart et al., 2021
Baboon	MACSFACS sorting (> 95%) CD4^+^CD25^*hi*^	1.7% spleen, 3.1% lymph node, 1.9% blood T cells; 10 × 10^4^ cells/ml blood	Pig PBMC^+^ IL-2; 3–4 week + 7–10 days without PBMC	≤ 2,000-fold, depending on IL-2 concentration	1:1^*a*^, strong xenogeneic suppression, donor-specific: 4–10 x less efficient to third-party	Porter et al., 2007
Baboon	CD4^+^CD25^*hi*^FACS-sorted from PBMC (> 95% purity)	1–2% of CD4^+^ cells	Stimulation with irradiated pig PBMC or anti-CD3/CD28 in cultures supplemented with IL-2 and rapamycin for 4 weeks	200-fold	Suppression of autologous anti-pig T effector cell and B cell proliferation	Singh A. K. et al., 2012
Baboon	FACS CD4^+^CD25^*hi*^ (top 1% of CD25^+^ cells) from PBMC	10^5^ Treg isolated from 20 ml blood	Culture for 26 days with IL-2, anti-CD3 Ab, aAPCs (transfected with human CD58, CD32, and CD80) and rapamycin, with weekly restimulation	>10,000-fold	Excellent suppressive function,. preserved or even enhanced by increasing amounts of restimulation after thawing	Weiner et al., 2015
Baboon	CD4^+^ T cells	n/a	Stimulation with tolerogenic, baboon Mo-derived DCs loaded with porcine-specific *in vitro*-transcribed RNA in cocultures supplemented with IL-2 and rapamycin for 10 days	Fivefold within 10 days	Highly suppressive effects on porcine-specific T effector cell proliferation; reduced IFNg/enhanced IL-10/TGFb production	Li et al., 2018

*(a)APC, (artificial) antigen-presenting cell; BM-DC, bone-marrow derived dendritic cells; CD40L-sBc, CD40 ligand-stimulated B cells; CFSE-MLR, carboxyfluorescein succinimidyl ester-mixed leukocyte reaction; FACS, fluorescence-activated cell sorting; LN, lymph node; MACS, magnetic-activated cell sorting; Mo-derived DC, monocyte-derived dendritic cells; MS, multiple sclerosis; TGFb, transforming growth factor b.*

Weiner et al. (2015) flow-sorted CD4^+^CD25^*hi*^ cells from baboon PBMC, followed by expansion with IL-2, anti-CD3 Ab, aAPCs (transfected with human CD58, CD32, and CD80), and rapamycin, with weekly restimulation. Expanded Treg were cryopreserved for 2 months, after which they were thawed and cultured for 48 h with the same stimulating agents. The purified Treg were expanded > 10,000-fold and exhibited excellent suppressive function. Cryopreservation reduced the cells’ suppressive function without changing their phenotype, but increasing levels of reactivation post-thawing improved cell viability and function, with a shift toward greater Treg purity. Thus, both the phenotype and function of the Tregs were preserved or even enhanced by increasing levels of restimulation post-thawing, reinforcing the concept of banking expanded recipient Tregs.

## Migratory Properties

Treg migratory ability is considered key to their *in vivo* homing to lymphoid tissues and sites of inflammation considered critical locations of their immunosuppressive function. While Treg markers are expressed in either accepted or rejected NHP kidney allografts (Haanstra et al., 2007), Treg recruitment to the interstitium of the graft has been implicated in metastable kidney transplant tolerance in rhesus macaques (Torrealba et al., 2004). Numerous studies, including those in transplanted animals (Chen and Bromberg, 2006; Lamarche and Levings, 2018; Mempel and Marangoni, 2019) have shown that the expression of specific chemokine receptors, integrins and selectins is required for Treg activity *in vivo* (Qin et al., 2008; Zhang et al., 2009) and that maximal graft protection occurs when Tregs migrate to both the transplant and the draining lymphoid tissue. Thus, optimization of procedures for generation of highly suppressive NHP Treg needs to include evaluation of the expression of a range of chemokine receptors compatible with their *in vivo* migration to both the allograft and lymphoid tissues. Zhang et al. (2015) reported that *ex vivo*-expanded polyclonal cynomolgus Treg expressed high levels of CXCR3/low levels of CD62L and CCR7, consistent with their potential accumulation at sites of inflammation.

## *In vivo* Mobilization and Depletion

The influence of cytokine and other biological agent administration on Treg in NHP has been investigated (Table 2). Thus, specific hematopoietic growth factors have been evaluated for their ability to selectively increase Treg *in vivo*, with potential to enhance their therapeutic efficacy, whereas Treg-selective depleting agents enable assessment of the dependency of tolerance-promoting protocols on these cells.

**TABLE 2:** Agents used to selectively enhance or deplete Tregs in NHP species.

Agent	Species	Dosage	Reported effect	References
**Enhancing agents**				
IL-2	Cynomolgus macaque	10^6^ IU/m^2^/day	Increased peripheral blood CD4 and CD8 Tregs (mainly CD45RA^–^ Foxp3^*hi*^)	Aoyama et al., 2012
IL-2	Rhesus macaque	10^6^ U/m^2^/day in combination with adoptively-transferred autologous Treg and rapamycin	Doubling of peripheral blood Treg compared with Treg infusion and rapamycin alone; stable expression of Treg gene transcripts	Furlan et al., 2020
IL-2	Cynomolgus macaque	0.6–3 × 10^6^ IU/m^2^	Acute cellular rejection of tolerated renal allografts 1–10 years post-transplant; reactivation and expansion of alloreactive T effector memory cells	Yamada et al., 2015
AMD3100 (Plerixafor),- antagonist of CXCR4 and CXCL12-mediated chemotaxis	Rhesus macaque	1 mg/kg (single dose)	CD4^+^/CD25^*hi*^CD127^*lo*^FoxP3^+^ Tregs mobilized efficiently using AMD3100-containing regimens; up to fourfold enrichment in leukapheresis products compared with use of G-CSF alone	Kean et al., 2011
GM-CSF and G-CSF	Rhesus macaque	GM-CSF (Leukine; 10 μg/kg/day); G-CSF (Neupogen; 10 μg/kg/day)	Significant elevation of Treg in peripheral blood and leukapheresis products	Sasaki et al., 2020
**Depleting agents**				
IL-2-diphtheria toxin fusion protein	Cynomolgus macaque	Two doses (8 or 18 μg/kg)	Rapid, but short-lived decrease in peripheral blood resting Tregs (CD4^+^CD45RA^+^Foxp3^+^) with a transient increase in activated Tregs (CD4^+^CD45RA^–^Foxp3^*hi*^), followed by their depletion by50–60%	Yamada et al., 2012b
Anti-human CCR4 immunotoxin	Cynomolgus macaque	25 mg/kg twice a day for four consecutive days, 6 h apart	78–89% CCR4^+^Foxp3^+^ Treg reduction in peripheral blood for approx 10 days; 89–96% CCR4^+^Foxp3^+^ Treg depletion in lymph nodes	Wang et al., 2016

**G(M)-CSF, granulocyte (macrophage)-stimulating factor.**

### IL-2

Inoculation of low dose IL-2 (10^5^–5 × 10^6^ IU/m^2^) expands CD4^+^Foxp3^+^ Tregs preferentially due to the cells’ expression of the high affinity IL-2 receptor alpha chain (CD25) (Zorn et al., 2006; Sakaguchi et al., 2008; Liao et al., 2013). Aoyama et al. (2012) reported that administration of low-dose IL-2 (1 million international units/m^2^ BSA/day) significantly expanded peripheral blood CD4^+^ and CD8^+^Tregs in normal cynomolgus macaques, with restricted expansion of non-Tregs. The expanded Tregs were principally CD45RA^–^ Foxp3^*hi*^ activated Tregs, with strong immunosuppressive activity *in vitro*.

Exposure of Treg to high IL-2 concentrations during their expansion can render the cells sensitive to “cytokine withdrawal–induced death” (Larsen et al., 2017) following their adoptive transfer. This phenomenon could potentially be alleviated by systemic IL-2 administration. Thus, Furlan et al. (2020) found that, in non-transplanted monkeys, adding low dose IL-2 (1 million units/m^2^/day) to rapamycin *in vivo* (target trough level: 5–15 ng/ml) promoted a logarithmic increase in the half-life/persistence of adoptively-transferred, autologous NHP Treg, in effect doubling the number of stable circulating Treg compared with Treg infusion in combination with rapamycin alone.

Yamada et al. (2015) examined the influence of systemic IL-2 on T cell alloreactivity and the maintenance of tolerance to MHC mis-matched kidney allografts induced in cynomolgus macaques via mixed hematopoietic cell chimerism. When given low doses of IL-2 (0.6–3 × 10^6^ IU/m^2^), animals that had accepted their grafts for 1–10 years in the absence of IS rejected acutely, with reactivation/expansion of alloreactive effector memory T cells. After stopping IL-2 administration, graft rejection was reversed and normal renal function restored.

### Hematopoietic Growth Factors

Kean et al. (2011) found that a small molecule antagonist of CXCR4- and CXCL12-mediated chemotaxis (AMD3100; Plerixafor) mobilized circulating lymphocytes in rhesus macaques, with significant increases in Tregs. CD4^+^CD25^*hi*^CD127^*lo*^FoxP3^+^ Tregs were mobilized efficiently, with increases as great as fourfold in leukapheresis products when compared with G-CSF administration alone. Overall, the results indicated that AMD3100 could mobilize a T cell repertoire that might provide protection against GVHD, and thus be of potential benefit in allogeneic hematopoietic stem cell transplantation. Also, in rhesus macaques, Sasaki et al. (2020) observed that combining GM-CSF and G-CSF administration increased the incidence of Treg in both blood and leukapheresis products. In these studies, the mobilized Treg exhibited a similar range of transcription factors, surface markers and chemokine receptors to Treg in normal monkey peripheral blood Treg. Moreover, when the mobilized Treg were expanded *ex vivo*, they displayed similar capacity to inhibit autologous CD4^+^ and CD8^+^ T cell proliferation.

### Depletion of Treg

Intravenous injection of cynomolgus monkeys with two doses of an IL-2-diphtheria toxin fusion protein (denileukin diftitox; 8 or 18 μg/kg) resulted in a rapid, but short- duration reduction in circulating resting Tregs (CD4^+^CD45RA^+^Foxp3^+^) accompanied by a transient elevation in activated Tregs (CD4^+^CD45RA^–^Foxp3^*hi*^), followed by their partial depletion (50–60%) (Yamada et al., 2012a). Wang et al. (2016) demonstrated that an anti-human CCR4 immunotoxin bound and depleted cynomolgus CCR4^+^ cells *in vitro*. In addition, they showed that the immunotoxin bound to the CCR4^+^Foxp3^+^ monkey Tregs *in vitro*. *In vivo* studies carried out in two naive cynomolgus revealed 78–89% CCR4^+^Foxp3^+^ Treg depletion in the peripheral blood that lasted about 10 days. In lymph nodes (LN), 89–96% CCR4^+^Foxp3^+^ Tregs were depleted. However, no effect was observed on other immune cell populations, including other CD4^+^ cells, CD8^+^ T cells, B cells and NK cells.

## Influence of Is Regimens on Treg in Allograft Recipients

The existence of Treg in NHP kidney allografts during their rejection has been considered integral to the rejection response (Haanstra et al., 2007). On the other hand, specific induction of Tregs by donor Ags and intragraft enrichment of Tregs may be key to long-lasting tolerance in NHP induced by transient mixed chimerism (Hotta et al., 2016; Matsunami et al., 2019). Co-stimulation blockade (Co-SB) of the CD28 pathway is deleterious to Treg function, due likely to the importance of the complimentary CTLA4-CD80/86 pathway in Treg development and homeostasis. Thus, administration of CTLA4-Ig (Abatacept) decreases circulating Tregs in MHC-mismatched rhesus renal transplant recipients (Anderson et al., 2019). However, Poirier et al. (2015) found that a novel antagonistic pegylated anti-CD28 Fab’ Ab fragment (FR104), together with low dose tacrolimus or rapamycin in a steroid-free treatment regimen, prevented acute allograft rejection and alloAb development, with accumulation of Helios^–^ Tregs in the blood and graft. Blocking CD28 using a monovalent, non-activating single chain anti-CD28 Fv fragment linked to alpha-1 anti-trypsin (sc28AT) synergized with CNI in cynomolgus kidney and heart transplantation, increasing absolute numbers of peripheral Tregs (Zhang et al., 2018). Kim et al. (2017) found that a novel anti-human CD40L (CD154) domain Ab (dAb) that prolonged rhesus renal allograft survival without thromboembolism, and that synergized with conventional IS to more markedly control graft rejection, increased CD4^+^CD25^+^Foxp3^+^ Treg frequency.

Ezzelarab et al. (2013, 2018) reported that infusion of donor-derived DCreg 1 week before transplant prolonged rhesus renal allograft survival in combination with CD28 Co-SB and rapamycin and promoted maintenance of donor-reactive CD4^+^CTLA4^*hi*^ Tregs.

## Treg Therapeutic Protocols in Transplant Recipients

Successful development of a therapeutic protocol based on adoptive transfer of Treg must address: (i) Treg efficacy and the number of cells required to achieve a therapeutic effect; (ii) stability of the suppressive phenotype; (iii) the Treg migratory pattern that assures their optimal regulatory function; (iv) the Ag specificity required for safe/effective control of rejection; (v) the impact of lymphocyte depletion/concomitant IS therapy on Treg function and durable control of rejection; (vi) conditions permissive to regulation of memory T cell responses. Several NHP studies (Table 3) have assessed feasibility, safety and therapeutic efficacy of adoptively-transferred, autologous Treg in transplant recipients. In a direct comparison of the persistence of transferred autologous vs. allogeneic Treg in peripheral blood of immunosuppressed, but not transplanted cynomolgus, we found that autologous Tregs survived much longer than the former (Zhang et al., 2015), a property suggesting more durable potential efficacy of autologous Tregs.

**TABLE 3:** Assessment of adoptive Treg therapy in NHP transplant recipients.

Type of graft (species)	IS therapy/conditioning	Type of Tregs (number/infusions)	Result	References
Kidney (rhesus) *n* = 6	Cyclosporine and post-transplant cyclophosphamide	Autologous splenocyte-derived “suppressive T cells” (approx 10^7/^kg) rendered anergic following co-culture with donor alloAg and anti-CD80/86 mAbs (10^2^ ± 67 × 10^6^ total on day 13 post-transplant)	Donor-specific tolerance in 50% of graft recipients	Bashuda et al., 2005
Kidney (cynomolgus) *n* = 4	ATG and low dose rapamycin	Expanded, donor Ag-specific, host splenocyte–derived CD4^+^CD25^+^Treg (14 daily infusions; 10^7^per day)	Graft MST prolonged from 22 to 48.5 days	Ma et al., 2011
Kidney (cynomolgus) (*n* = 5)	Non-myeloablative conditioning and MHC-mismatched BMT. Renal transplantation (from the same BMT donor) conducted 4 months after BMT, with no IS	Expanded polyclonal autologous Treg (15–53 × 10^6^/infusion) during the 1st week post-transplant (days 0, 2, 5, 7) and day + 50 (total dose: 88–96 × 10^6^/kg)	Two of 5 evaluable recipients of Treg + BMT displayed T cell chimerism up to 335 days post-BMT. In one long-term surviving animal, the delayed kidney graft survived > 294 days without IS, however, non-Treg BMT recipients rejected their delayed kidney grafts within 3–4 weeks	Duran-Struuck et al., 2017
Heart (cynomolgus) *n* = 5	ATG, tacrolimus, anti-IL-6R mAb and tapered rapamycin maintenance IS therapy	Expanded polyclonal Tregs (single or multiple doses (up to a maximum cumulative cell dose of 1.87 billion cells during the early post-transplant period (up to 1 month post-transplant)	Inferior graft function with multiple infusions; elevated incidences of T effector memory cells, increased IFNγ production by host CD8^+^ T cells, enhanced levels of proinflammatory cytokines and anti-donor alloAb	Ezzelarab et al., 2016
Heart (cynomolgus) *n* = 5	ATG, tacrolimus and anti-IL-6R with tacrolimus conversion to rapamycin at 2 weeks (early cell infusion within 3 weeks post-transplant); ATG and tacrolimus with tacrolimus conversion to rapamycin at 2.5 weeks (delayed cell infusion, 6–8 weeks post-transplant)	Expanded donor Ag alloreactive Tregs; 20.5–120 × 10^6^/kg for each of 2–4 infusions	No prolongation of graft survival; loss of regulatory signature and proliferative/survival capacity by transferred Tregs	Ezzelarab et al., 2020
Pig pancreatic islets (xeno; rhesus) *n* = 3	ATG, CVF, anti-CD154 mAb, and rapamycin	Intraportal infusion (x1 or x2) of expanded CD4^+^CD25^*hi*^CD127^*lo*^ autologous Tregs (1.87–62.0 × 10^6^) following ATG depletion	Treg infusion associated with more stable and durable normoglycemia	Shin et al., 2015
Pig pancreatic islets (xeno; rhesus) *n* = 2	ATG, CVF, anti-CD154 mAb and rapamycin	As above (ref 65)	Engrafted pig islets rejected by activated T cells following withdrawal of maintenance IS	Shin et al., 2016
Pig skin graft (xeno; baboon) *n* = 4	Splenectomy, TBI, ATG, TI, rapamycin, CVF, GalKO/huCD46/huCD47 transgenic donor pig HSCs, anti-CD40LAb, methylprednisolone	25 × 10^6^/kg (8 infusions)	Prolonged donor skin graft acceptance	Stern et al., 2017

**ATG, anti-thymocyte globulin; BMT, bone marrow transplantation; CVF, cobra venom factor; Gal KO, α1,3-galactosyltransferase gene-knockout; HSCs, hematopoietic stem cells; hu, human; IS, immunosuppression; MST, mean/median graft survival time; TBI, total body irradiation; TI, thymic irradiation.**

### Renal Transplantation

The earliest work (Bashuda et al., 2005) was conducted in rhesus macaques given MHC-mismatched renal allografts. Thus, autologous spleen-derived “suppressive T cells” (approx 10^7/^kg) that were rendered anergic by co-culture with donor alloAg together with anti-CD80/CD86 mAbs were infused once, 13 days post-transplant to splenectomized hosts that receiving brief cyclosporine and cyclophosphamide (Cy) treatment. Grafts survived long-term and donor-specific tolerance was achieved in 50% of recipients (*n* = 6), but not in controls, confirming the potential of a Treg therapy in NHP organ transplantation. These findings provided the basis for a clinical trial in living donor liver transplantation, in which splenic T cells rendered anergic to donor and administered 13 days post-transplant after Cy, induced operational tolerance in 7/10 recipients (Todo et al., 2016). However, infusion of similarly generated Tregs 12 days post-transplant into living donor kidney transplant patients resulted in high rates of rejection upon subsequent IS drug withdrawal (Koyama et al., 2020).

Ma et al. (2011) reported that *ex vivo*-expanded autologous Treg prolonged renal transplant survival in ATG-treated cynomolgus monkeys. In this study, a much greater number of infusions (fourteen) of expanded, donor alloAg-specific, spleen–derived CD4^+^CD25^+^Treg were infused (10^7^ per day). The infusions started at the time of transplantation (i.e., 1 day following a 3-day course of ATG) and were administered together with low-dose rapamycin for 14 days. Thus, kidney graft survival was prolonged significantly, but unlike in the aforementioned study, no grafts survived indefinitely.

Duran-Struuck et al. (2017) reported that recipient Treg co-transfer could enhance bone marrow (BM) engraftment/hematopoietic cell chimerism and prevent cynomolgus kidney allograft rejection. Eight monkeys were subjected to non-myeloablative conditioning and MHC-mismatched BM transplantation (BMT), either with or without infusion of Treg. Transplantation (from the same BM donor) was undertaken 4 months post-BMT, in the absence of IS to evaluate robust, donor-specific tolerance. Five animals received *ex vivo*-expanded polyclonal autologous Treg during the first week post-transplant (days 0, 2, 5, 7) and also on day 50. Transient mixed chimerism, without significant T cell chimerism, was observed in those monkeys given BMT but no Treg (*n* = 3). By contrast, the 2 of 5 monkeys given Treg + BMT that could be evaluated showed multilineage (including T cell) chimerism up to 335 days after BMT. It was notable that, in the monkey that survived long-term, >90% of donor T cells were found to be new thymic emigrants. In this monkey, the delayed (to 4 months) renal transplant was accepted for >294 days without IS therapy, whereas non-Treg BMT recipients rejected their delayed kidney grafts within 3–4 weeks. Early reactivation of cytomegalovirus (CMV) and anti-viral treatment was linked with early failure of chimerism, irrespective of Treg administration. Overall, these observations reveal that, without early CMV reactivation (and consequent BM-toxic anti-viral therapy), administration of host Treg can promote both prolonged multilineage chimerism and robust donor tolerance.

### Heart Transplantation

Addressing the hypothesis that markedly reduced T cell numbers in graft recipients would favor the therapeutic efficacy of adoptively-transferred Tregs, Ezzelarab et al. (2016) infused *ex vivo*-expanded, polyclonal Treg into ATG-treated, MHC-mismatched cynomolgus monkey heart transplant recipients before the homeostatic recovery of effector T cells. Tacrolimus, anti-IL-6R mAb and tapered rapamycin maintenance treatment was also administered. Infusion of Treg in either single or multiple doses during the early post-transplant period (up to a month post-transplant) during which time host T cells were markedly depleted, resulted in poorer heart graft function compared with non-Treg-infused controls. This was accompanied by an increased incidence of circulating effector memory T cells, elevated IFNγ production by CD8^+^ T cells, and enhanced levels of circulating proinflammatory cytokines and anti-donor alloAb. These observations suggest that Treg infusion early post-transplant period following lymphodepletion should be avoided in human clinical trials. Thus, despite marked but transient increases in circulating Treg relative to effector T cells and the use of so-called “Treg-friendly” agents, environmental conditions and host immune effector mechanisms that prevail under these conditions may negate the potential therapeutic efficacy of the infused transferred Treg.

In a more recent study (Ezzelarab et al., 2020), cynomolgus monkey autologous darTreg were expanded from flow-sorted, circulating Treg using activated donor B lymphocytes and infused after transplant into MHC-mismatched heart graft recipients. While the darTreg selectively suppressed proliferative responses of autologous T cells to donor alloAgs *in vitro*, their adoptive transfer post-transplant failed to prolong graft survival. Early (within 2 weeks post-transplant; under ATG, tacrolimus and anti-IL-6R) or delayed (6–8 weeks post-transplant; under rapamycin) darTreg infusion resulted in a rapid reduction in transferred cells in the circulation. After early or delayed infusion, dye-labeled darTreg could be observed in lymphoid and non-lymphoid tissues and in the heart graft at low percentages (<4% CD4^+^ T cells). Notably, the infused darTreg displayed reduced expression of Foxp3, CTLA4, Helios, the proliferative marker Ki67, and anti-apoptotic Bcl2, compared with pre-infusion darTreg and endogenous Treg.

### Comparison of Doses of darTreg Tested in NHP and Human Allograft Recipients

Doses of darTreg tested in cynomolgus heart allograft recipients following lymphodepletion with ATG (Ezzelarab and Thomson, 2020) were similar to or greater than doses of autologous T cells rendered anergic to donor Ag and infused post-transplant to Cy-treated, renal-allografted monkeys (Bashuda et al., 2005) and that induced donor-specific tolerance. However, they also resemble the single doses of similarly generated Tregs (14–36 × 10^6^/kg) infused 12 days post-transplant to living donor kidney transplant patients, including those given Cy, that, by contrast, exhibited high rates of rejection upon subsequent IS drug withdrawal (Koyama et al., 2020). In other clinical studies of darTeg in living donor kidney transplantation, lower doses of darTreg have been targeted (i.e., 2 × 10^3^–2 × 10^6^/kg or 0.5–10 × 10^6^/kg, respectively) in small numbers of patients at separate centers in the ONE Study (Sawitzki et al., 2020) in which overall safety of cell therapy and similar 1-year graft survival compared to a reference standard of care group have been reported. In human living donor liver transplantation, doses of 23.3–14.4 × 10^6^ T cells rendered anergic to donor and administered 13 days post-transplant after Cy induced operational tolerance in 7/10 recipients (Todo et al., 2016). A total of 300–500 × 10^6^ darTreg have been targeted in a liver transplantation IS drug withdrawal study at UCSF (NCT02474199).

## Tracking/Monitoring of Polyclonal or Dartregs in Normal NHP or Organ Allograft Recipients

The *in vivo* persistence and migration of adoptively-transferred polyclonal Tregs to secondary lymphoid tissues documented in rodents have been confirmed by NHP studies that have determined the survival, migration, and function of exogenous Tregs. Detection of autologous or allogeneic Tregs infused into normal macaques has been accomplished by direct dye-labeling and subsequent tracking of the Tregs in blood, LNs and spleen at various times after their infusion (Singh et al., 2014; Zhang et al., 2015). Pharmacokinetic analysis of dye-labeled autologous Tregs has revealed an initial rapid period of elimination from the blood between day 0 and 3 post-infusion, after which the transferred Tregs persist at low levels for up to 3 weeks (Zhang et al., 2015). Staining for the cell proliferation marker Ki67 further demonstrates that label dilution as a result of cell proliferation does not contribute to the apparent disappearance of transferred Tregs from blood. Labeled autologous Tregs have been detected in LNs on day 1–2 post-infusion, however analysis on day 6 failed to demonstrate sustained persistence of infused Tregs in secondary lymphoid organs (Zhang et al., 2015).

Concurrent IS therapy markedly increases the survival of adoptively-transferred autologous Tregs in the peripheral blood and LNs. Labeled autologous Tregs persist longer in monkeys given rapamycin and in greater numbers compared to non-immunosuppressed conditions at least 50 days post-infusion (Furlan et al., 2020). Low dose IL-2 together with rapamycin further prolongs the half-life of adoptively-transferred Tregs in NHPs, with detection of labeled cells in the periphery up to 84 days after infusion. These findings highlight a wide variability in the survival of infused Tregs under different conditions, including the use and type of IS, in addition to cell production methods, including cryopreservation.

## Xenotransplantation

Treg in xenotransplantation has been reviewed (Ezzelarab, 2018). Baboon Treg expanded in response to irradiated pig PBMC for potential use in pig-to-baboon xenotransplantation (Porter et al., 2007) proved strongly suppressive *in vitro* and donor-specific suppression was achieved. Huang et al. (2017) found that baboon autologous Tregs expanded by stimulation with pig PBMC could prevent porcine islet xenograft rejection in NOD-SCID IL-2rγ^–/–^ mice reconstituted with baboon PBMC. Prolonged xenograft survival to >100 days correlated with Treg engraftment and intragraft CD39 and Foxp3 gene expression. Shin et al. (2016) transplanted two diabetic rhesus with pancreatic islets isolated from wild-type miniature pigs with IS comprising ATG, cobra venom factor, anti-CD154 mAb and sirolimus. Expanded CD4^+^CD25^*hi*^CD127^*lo*^ autologous Tregs were infused during the peri-transplant period, however following withdrawal of maintenance IS, engrafted pig islets were rejected, indicating failure of tolerance induction by the autologous Tregs in this model.

## Conclusion and Future Studies

NHP have the inherent advantage over rodent or humanized/primatized mouse models of closely resembling the human condition. Endogenous Treg in NHP can be increased or selectively depleted *in vivo*, and both polyclonal and darTreg have been expanded successfully *ex vivo*. In NHP kidney, heart and pancreatic islet transplantation, single or multiple infusions of autologous Treg have yielded results ranging from indefinite, IS-free graft survival to exacerbation of acute rejection, depending on the experimental model and IS regimen. In addition to valuable safety and graft outcome data that help guide clinical trial design, important insights have been gained into the biodistribution, stability and longevity of the transferred cells, and their influence on anti-donor immunity. These findings have drawn attention to the biological and logistical challenges encountered when transitioning testing of Treg therapeutic efficacy in inbred, spf mouse models, usually at very high/unphysiological Treg/effector cell ratios, to more clinically relevant NHP species. Exciting, newly evolving approaches to generation of stable, Ag-specific Tregs (Ferreira et al., 2019; Raffin et al., 2020), include gene editing of bulk T cells (Honaker et al., 2020) and production of CAR Tregs engineered to promote their Ag specificity and homing (MacDonald et al., 2016; Dawson et al., 2019; Hoeppli et al., 2019; Mohseni et al., 2020). Although there are no published reports of these developments as yet in NHP models, testing of such advances in NHP organ transplantation is keenly anticipated.

## Author Contributions

AT, KS, and ME participated in planning of the manuscript, literature searches, and in the writing of the mini-review. All authors contributed to the article and approved the submitted version.

## Conflict of Interest

The authors declare that the research was conducted in the absence of any commercial or financial relationships that could be construed as a potential conflict of interest.

## Abbreviations

Ab: antibody
Ag: antigen
(a)APC: (artificial) antigen-presenting cell
ATG: anti-thymocyte globulin
Co-SB: co-stimulation blockade
Cy: cyclophosphamide
darTreg: donor antigen alloreactive regulatory T cells
IS: immunosuppression/immunosuppressive
NHP: non-human primate
PBMC: peripheral blood mononuclear cells
spf: specific pathogen free
Teff: T effector cell(s)
TGF β: transforming growth factor β
Tmem: memory T cell(s)
Treg: regulatory T cell(s).
